The article "Application of Data Resource Allocation in Economic Management Information System" was published in 2022. Journal: Comput Intell Neurosci.

# Application of Data Resource Allocation in Economic Management Information System

**DOI:** 10.1155/2022/1346646

**Published:** 2022-05-11

**Authors:** Yi Guan, Qian Chen, Zhilin Li

**Affiliations:** ^1^College of Information and Business Management, Dalian Neusoft University of Information, Dalian 116023, Liaoning, China; ^2^School of Logistics Management and Engineering, Zhuhai College of Science and Technology, Zhuhai 519041, Guangdong, China

## Abstract

With the development of the digital economy and the sharp increase in economic information, a large amount of data needs to be processed. Therefore, the demand for an economic management information system is also increasing, but how to realize the allocation of data resources in the system has become an urgent problem to be solved. This study conducts research on the above problems, first analyzes the research results of domestic and foreign scholars, finds out the content suitable for this research, and then introduces the structure of the economic management information system and the method of data resource allocation in detail. Finally, by comparing and testing the algorithm of data resource allocation and other allocation algorithms, it is concluded that the allocation algorithm used in this study is more effective than the research algorithm of previous scholars, thus proving the feasibility of this research. The test results show that the number of protocol function modules allocated by the GAA algorithm is 20% to 30% less than that of the RAA algorithm. So, it can be concluded that compared with the RAA algorithm, the GAA algorithm saves more network resources.

## 1. Introduction

In recent years, the macroeconomic situation at home and abroad has become increasingly complex and severe. The international economic downturn and domestic difficulties have been superimposed on each other, resulting in unstable and uncertain factors in economic operation. Under such circumstances, how to accurately judge the economic situation and take effective measures in a timely manner is more important. Therefore, it is very necessary and urgent to promote the construction of macroeconomic management information system engineering. This makes macroeconomic research increasingly important, importance of this to macroeconomic research has become increasingly prominent, and the project management of macroeconomic management information systems also has a positive role in promoting the analysis of macroeconomic-related information.

As the number of communication users increases and people's demands for services increase, traditional mobile communication systems are becoming more and more difficult to meet the diverse service demands of users. The closed networking mode and static configuration management mode will cause many problems such as uneven distribution of system resources and degraded user experience. SDN adopts a centralized control mode, which separates the management and control functions of virtual networks from physical devices by means of network software definition, so that flexible programming and modification can be realized according to business requirements to improve the level of network intelligence. In an SDN network, network managers dynamically allocate network resources according to business requirements. Therefore, the research work on the SDN network resource allocation method is crucial.

The innovation of this study is that

1. Compared with previous research work, most of the controller deployment schemes based on software-defined networking (SDN) are considered from the perspectives of reducing propagation delay, load balancing between controllers, and improving reliability. This study focuses on the problem of signaling overhead between controllers when users receive management from different controllers in the process of frequent random movement. Taking the user's moving behavior as the similarity, the spectral clustering algorithm is used to implement the controller deployment.
2. Since the total number of protocol function blocks is reduced, the network can save a lot of transmission computing resources for other service flows, thereby improving the overall resource utilization of the network. Therefore, on this basis, this study focuses on how to allocate the minimum number of protocol function modules to each type of request in a time-limited network.
3. This study takes the macroeconomic management information system project management as the research object, firstly summarizes the theory related to project management, then gives a brief overview of the macroeconomic management information system, and then analyzes the various elements of the macroeconomic management information system on this basis. By expounding the human resource management, risk management, and communication management of this system development project, the value of the whole project is finally concluded.

## 2. Related Work

Regarding the research on economic management information system and data resource allocation, many scholars at home and abroad have provided a lot of references.

Wan proposed an ontology-based resource reconstruction method. First, the Web Ontology Language (OWL) is used to build the intelligent device ontology that describes the intelligent manufacturing resources. On this basis, the relational database is associated with the manufacturing system ontology, so that the manufacturing resources are mapped to the model instance. Finally, taking the intelligent manipulator device reconfiguration as an application case, the proposed ontology-based resource reconfiguration method is expounded, and its feasibility in manufacturing is verified [1].

Zhang proposed a new energy consumption model that considers random workloads of VMs that support reconfiguration of computing power. Without specifying any workload distribution, Zhang proves that there is theoretically an optimal SRP that achieves the minimum energy cost, and Zhang derives a closed form of the conditions for achieving this minimum energy point. Zhang also derives a closed form for computing the optimal SRP when the workload follows a Gaussian distribution. Then, Zhang studies the joint workload distribution and computation frequency configuration problems for multiple distributed VM scenarios and proposes solutions to the Gaussian distribution and unspecified distribution problems. The performance evaluation results by Zhang on synthetic and real workload tracking data demonstrate the effectiveness of the proposed model. The closeness of the simulation results to the analysis results proves that the method proposed by Zhang can achieve lower energy consumption compared with the fixed computing power allocation method [2].

Yao evaluated the impact of free space optic (FSO) links on inter-rack (IRS) networks. Evaluation results show that the FSO link reduces the average number of communication hops for user jobs, approaching the best possible value of 2 hops, thus providing benchmark performance comparable to the corresponding rack-level architecture. Furthermore, if four FSO terminals are allowed per rack, the CPU/SSD (GPU) interconnect latency is 25.99% lower than fat tree and 67.14% lower than 2D Torus. Yao also demonstrated the advantages of an FSO-equipped IRS system in terms of the average turnaround time of scheduled jobs given a set of benchmark workloads [3].

Vokeman explores whether the relationship between teachers' person-organization (P-O) fit, job satisfaction, and transfer intention differs depending on how a range of human resource (HR) practices is configured in education [4].

Dharan explores the evolution from basic classic “isolated” legacy infrastructure to on-premise modern data centers (DCs). The composable infrastructure proposed by Dharan B supports a variety of traditional and modern workloads, with flow pools of independent resource configurations [5].

Lee aims to improve performance (e.g., manufacturing time and job completion time for multiple jobs) without modifying the framework or application and avoid the problems of previous self-tuning approaches based on performance models or resource usage [6].

The data of these studies are not comprehensive, and the results of the studies are still open to question, so they cannot be recognized by the public and thus cannot be popularized and applied.

## 3. Economic Management Information System and Data Resource Allocation

### 3.1. Economic Management Information System

The continuous improvement of scientific, democratized, and legalized degree has put forward new requirements for the construction of macroeconomic management information system [7, 8].

(1) Supporting strong macroeconomic management information function. The system should include the following:
  1. Establishing a macroeconomic information database that meets the requirements of big data
  2. The rapid access and transmission of information are the general trend
  3. Using modern information technology and other multidisciplinary scientific knowledge to strengthen the analysis of macroeconomic information, realize the digitization of the macroeconomic management process, establish an information analysis system for macroeconomic management, and provide good support for macroeconomic control [9, 10]
(2) It can play a role in auxiliary analysis for decision-making. According to the needs of economic development, various economic analysis methods and tools are used to establish a corresponding decision-making system [11].
(3) It can better serve social development. To meet the requirements of the continuous progress of China's democratization, it is necessary to establish a democratic decision-making support system based on an extensive analysis of public opinion [12, 13].

The application requirements of this system mainly include the following four aspects: realizing the information sharing and sharing mechanism between various economic management departments and providing real-time and accurate economic data for the healthy development of the whole province's macroeconomy; improving the informatization level of economic management and improving the efficiency of economic management of the whole society; building a decision-making support system for macroeconomic and social management and regulation and enhancing the accuracy and effectiveness of economic decision-making; and, at the same time, enhancing the service and information release for the whole society [14].

#### 3.1.1. Sharing of Economic Information (as Shown in Figure 1)

Economic and social management requires comprehensive information support from big data. The most important thing is to improve the efficiency of information collection and analysis, and the need to realize information sharing and sharing among various economic sectors in society is becoming more and more urgent [15, 16].

#### 3.1.2. Big Data in Economic Management

Economic management is the main link of macroeconomic management, which has the characteristics of wide coverage, complexity, and high requirements. The big dataization of business management is a new requirement in the Internet era [17]. A schematic diagram of the business management informatization process is shown in Figure 2.

#### 3.1.3. Auxiliary Decision Support

With the increasing complexity of economic development, the level of economic management in the industry is also getting higher and higher. The previous effective decision-making methods and means have been inappropriate, and a new decision-making support system and process need to be established [18, 19]. A schematic diagram of the economic decision-making process is shown in Figure 3.

#### 3.1.4. The Coordination Work Is Heavy

To ensure the realization of the macroeconomic management goals of A Province, policy coordination and business coordination must be carried out between different departments and different businesses, and the construction of a new decision-making support system provides an excellent opportunity to resolve various conflicts in the new era [20]. A schematic diagram of policy coordination and business collaboration is shown in Figure 4.

The economic management information system should have the following basic functions:

1. Information Sharing: information sharing can provide specific and detailed services such as information inquiry for economic management functional departments and personnel [21, 22]
2. Big Data in Business Processing: using Internet computer technology to organize business processes, gradually realize the precision of economic management work, and meet the ability of economic management departments to analyze information in the Internet environment [23]
3. Decision Support: providing various models and tools required for economic analysis to meet the needs of various functional analysis under the new economic situation
4. Social Service: through the construction of the portal website, we can understand the voice of the whole society and the needs of ordinary people
5. Information Confidentiality: strengthening information security and confidentiality

At present, the economic management information system still has the following problems: there is no overall plan; it is difficult to integrate resources; it is difficult to communicate and coordinate among various departments; the business development is unbalanced; and the system construction is not sufficient to meet the needs.

The overall goal of this economic management information system is to rely on the e-government network platform of XX Province and realize the coordination and sharing of various economic management departments through the construction of information database, information sharing and sharing system, and application system construction of various key departments of economic and social management.

The software architecture of the economic management information system in XX Province follows the service-oriented architecture (SOA) idea and is designed in combination with cloud computing technologies and concepts. The overall architecture mainly includes data resource service layer, platform software service layer, and business software service layer. The data center provides IT infrastructure, network and information security, operation and maintenance management, and other services for the stable and safe operation of business software. The basic support resource configuration list is shown in Table 1.

The system framework consists of the following layers:

*(1). Data Layer*. This layer includes the configuration data of the portal and the data resources of the business system. Through the unified collection, exchange, and integration of data, a thematic database of economic topics is formed.

*(2). Business Layer*. This layer is a collection of business logic that supports applications in various departments. It sorts and integrates business through the service bus. The business layer connects the existing service operations, describes them uniformly into a business process according to specific rules, arranges and combines fine-grained services into different business processes (coarse-grained services), and realizes dynamization. Also deployed in the business layer is a BPEL workflow engine that is responsible for consuming services in sequence or necessary logic. The external system interface completes the docking with other information systems in XX Province (such as enterprise basic information sharing platform, other government affairs systems) and relevant national platforms. This docking utilizes the extensive connectivity of ESB and is realized in the form of services.

*(3). Presentation Layer*. This layer is composed of the economic management information system portal of XX Province. Through technical means such as interface integration, it realizes the unified management of users, the unified display of business, and the unified entrance of transaction processing, to meet the needs of the government, enterprises, and the public for economic information services.

The database is an important part of this economic management system design, and its data mainly come from various economic management departments and business application systems. According to the unified catalogue of information resources, a shared database of national economic and social development planning and planning, rural economy, macroeconomics, etc., is established, and a shared library of price policy documents mainly stores unstructured information. These shared databases are updated and maintained by each information collection channel and business application system established by this project. The calculation table of the computing power of the database server is shown in Table 2.

The information content of each database is as follows:

1. The rural economic database includes the rural economic planning plan database, the agricultural situation monitoring database, the rural economic statistics database, the rural price policy document database, the food security early warning database, and the expert knowledge base
2. The important commodity price database consists of the domestic market price database of important commodities, the government-priced commodity and service price database, the international market price database of important commodities, the import and export commodity price database, price policy documents, and thematic analysis databases
3. The macroeconomic database includes macroeconomic statistics, economic research, and policies and regulations
4. The fixed asset investment project database includes basic project information, investment information, owner information, and approval information

### 3.2. Design Principles of Business Database Design

The design of the application database of the macroeconomic management information system of XX Province is guided by the needs of economic management-related content, and it realizes the multidirectional collection and structural arrangement of data and provides data support for the macroeconomic management information system of XX Province. The calculation table of the computing power of the application server is shown in Table 3.

(2) Leading technology and good completion. It fully reflects technology leadership and technology development orientation and adopts industry-leading technology in technical specifications, product selection, and design methods; at the same time, it fully considers the requirements of planning and economic management for database security and reliability and selects mature technical products when selecting technologies.
(3) The information is comprehensive and standardized. By adopting data auditing and restraint mechanisms, the data are guaranteed to be comprehensive. The database design should not only consider a moderate margin but also ensure that the relevant data query is optimized. The normalization of the relational data model is adopted, and the degree of normalization is high.
(4) Ensure security and system scalability. It fully considers the confidentiality of the province's economic data, introduces authentication and authorization mechanisms, proposes data access security, and prevents illegal data access, data destruction, and data leakage; it fully considers the scalability of the macroeconomic management information system in XX Province, ensures that the database structure design is scalable, reserves a moderate margin in the design, and reserves space and interfaces for the expansion and migration of the macroeconomic management database.

#### 3.2.1. National Economic Development Planning Database

The construction of the national economic development planning shared database will establish a national economic development planning and planning index system, integrate data such as planning plans, investment projects, and comprehensive information on grain and oil, and build a database structure for national economic development planning plans.

By extracting relevant information from the business system in real time according to the standard of the shared database or entering it manually, it provides the data basis for the system to realize the analysis functions such as data loading, statistical summary, query, and retrieval.

#### 3.2.2. Rural Economic Management Database

The data source of the rural economic management shared database is the rural economic management information system and related departments. To support the business of this system, massive amounts of external data need to be informatized. Meanwhile, the rural economic management information system will generate a large amount of information in the process of processing business processes such as planning and economic situation analysis. Therefore, it is necessary to build a series of business databases in the rural economic management information system.

#### 3.2.3. Price Supervision Database

When the price supervision information system deals with the price management business process, firstly, it will generate massive internal data, and, secondly, it needs massive external data, and both require standardized information processing, so it is necessary to build a series of business databases.

#### 3.2.4. Fixed Asset Investment Project Management Shared Database

The fixed asset investment project management information system serves as an information platform for fixed asset investment planning, management, monitoring, and adjustment. The data generated by the system, including project approval, capital arrangement, dynamic monitoring and inspection, project filing, and decision support, are all included in this database for management. It mainly collects relevant data generated during the entire life cycle of fixed asset investment projects. The database includes the project database, project material library, and sub-libraries such as policy and regulation literature library.

The specific data include the following: the project approval system examines the basic information of the project, construction scale, benefits, and other information; issues the data of the capital arrangement plan, dynamic monitoring, and inspection; and regularly tracks the data of its implementation, the availability of funds, and the completion of investment and construction.

#### 3.2.5. Macroeconomic Monitoring and Early Warning Shared Database

The data source of the macroeconomic monitoring and early warning shared database is the macroeconomic monitoring and early warning system.

The monitoring data, early warning model data, calculation results, and early warning data required for system operation are all data content, including economic growth, economic momentum, price changes, employment changes, fiscal revenue, economic benefits, economic benefits of industries above designated size, comparison of the average annual growth of labor input and actual labor input, comparison of the average annual growth of total capital stock and production capital stock, distribution coefficient of domestically generated net value, contribution of total factor productivity improvement to economic growth, comparison of industrial specialization coefficient and social cooperation degree among provinces, municipalities and districts across the country, data on the change trajectory of the social cooperation degree of various industrial sectors in China, and the change trajectory of the social cooperation degree in the whole country and each province, city, and district.

#### 3.2.6. Energy Saving and Carbon Reduction Database

The data source of the energy-saving and carbon reduction database is the energy-saving integrated information management system. The basis of system operation is the collection of energy information content, which is the fundamental and core content of database construction.

The construction of information resource database mainly realizes the collection, filtering, and classification of information content and enables users to query and browse the content in the process of data interaction.

The construction content of the comprehensive energy conservation database mainly includes eight sub-databases: energy conservation assessment of fixed asset investment projects, industrial energy conservation, building energy conservation, transportation, energy conservation assessment, energy conservation statistics, energy conservation monitoring, and resource and energy consumption of public institutions. The data come from different authorities.

### 3.3. Data Resource Configuration

The data resource configuration in this study is implemented using software-defined network architecture. Software-defined networking (SDN) emerged from OTT (Google B4 Traffic Engineering).  Figure 5 is a network architecture diagram of SDN. ONF defines SDN as a new network architecture that separates the control and forwarding functions of traditional networks and controls network behavior through programming. This new network architecture transforms the control function of the network from the underlying device to the outer computing device. The underlying device is abstract and transparent relative to the network application, enabling the virtualization of the network to be realized. The SDN controller deployment summary is shown in Table 4.

SDN has the following characteristics.

#### 3.3.1. Separation of Control and Forwarding

From the perspective of network architecture, SDN decouples the control plane and forwarding plane of the network, so that the control function of the network is no longer integrated into the network equipment. This closed way of fully releasing the control function from the network equipment and breaking the traditional integration of forwarding and control solves many problems existing in the traditional network and fully releases the network potential of SDN.

#### 3.3.2. Separation of Software and Hardware

In the future direction of network development, network equipment is gradually evolving toward a modular, standard, and transparent way, and the separation of software and hardware will become a future development trend. In SDN technology, the control function is separated from the network equipment and runs in the general server in software programming mode. This further simplifies the network hardware function, and the device also develops toward the general-purpose commercial hardware (commercial off-the-shelf, COTS). In NFV technology similar to SDN, the separation of software and hardware is more thorough, and network functions are implemented in software.

#### 3.3.3. Separation of Business and Network

SDN technology realizes the separation of business and network. The network controller only needs to define the corresponding business requirements. The specific network resource configuration methods, such as QoS, underlying device forwarding routing, and bandwidth allocation, are dynamically generated by the upper layer according to the business, and the controller realizes the data forwarding process of the underlying device.

#### 3.3.4. Open System Architecture

The open architecture makes the SDN network highly portable and compatible. It is mainly reflected in the following aspects: (a) the network architecture is open. The SDN architecture is a layered structure that separates the control and forwarding planes. There are corresponding standardized communication protocols between each layer, and standard interfaces are used for communication between different layers. (b) The core components are open. The open embodiment of SDN core components now allows external programming control, so that network entities can be dynamically deployed according to people's needs to achieve intelligent control. (c) Interfaces and protocols are open. SDN realizes the expansion of different applications in different network environments through the northbound interface, and SDN realizes the manipulation and scheduling of the underlying equipment according to different applications through the southbound interface.

#### 3.3.5. Centralized Control

There are two commonly used control methods: distributed control and centralized control. SDN technology adopts the latter. The advantage of this centralized control is that the SDN controller has a view of the entire network and has a global understanding of the network. The network manager can globally optimize the network according to different business requirements, thereby improving network performance and optimizing network resource allocation.

#### 3.3.6. User Programmable

The essence of SDN technology is that network managers can influence and modify network behavior in a standard programming way. According to the different requirements of the application layer, the underlying devices are controlled programmatically. The user-programmable function relies on the standard and unified network interface opened by SDN to the outside world.

#### 3.3.7. Forwarding Plane Abstraction

The abstraction of the forwarding plane is mainly reflected in the forwarding function of the underlying device. The underlying device only forwards data according to the instructions of the SDN and does not need to deal with other network protocols. In general, in the SDN architecture, for the application layer and the control layer, the bottom layer is equivalent to a logical switch with a forwarding function, which simplifies the complexity of the network, facilitates new service updates, and improves the flexibility of the network.

Based on the concepts and characteristics of SDN introduced above, this study will elaborate on each layer of the SDN network architecture.

Figure 6 is the detailed system framework of SDN. Next, each layer of the SDN architecture will be explained in detail, and the technology of each layer expansion will be introduced accordingly.

### 3.4. Application Layer

This layer is at the top of the SDN architecture. Based on the open network capability of the northbound interface of the controller, the network operator brings infinite possibilities to the application of SDN by flexibly programming the network, for example, combining new Internet applications such as cloud computing, big data, and the Internet of things to enhance network value; innovating network applications to improve network value-added service capabilities; realizing customized customization and improving user experience; according to the network operation situation, flexibly allocating network resources to optimize the utilization of network resources, improving network visualization, and realizing accurate, efficient and intuitive network operation, maintenance, and management.

In the application layer, the most important is the network orchestration technology. Network orchestration refers to arranging and organizing different logical service network units in a certain order according to different business requirements and adding controllers to form physical network services that meet user business requirements.

The process of network orchestration technology can be summarized as follows: business personnel define the business system and output the business template, and then, the network orchestration system maps out the logical network service view according to the template. The network view is an intermediate product, which does not involve the specific resource allocation process, but only converts the connection relationship of the components of the business system into the connection relationship of the network functional components and then abstracts the corresponding network model. For example, connection components such as L2, L3, VPN, and other flow-based network connection nodes and links are provided by switches, routers, and links; service components such as NAT, DNS, AAA, and other IP services are provided by corresponding service network elements. The above network functions will eventually be mapped to corresponding network entity devices in some form. After the network service view is formed, the orchestration system assigns tenant IDs to tenants according to different services, tenant information, and constraints to form a tenant logical network. Finally, the orchestration system sends the tenant's logical network to the controller through the northbound interface. The controller is then mapped to the corresponding physical network, and the devices at the data layer are configured and implemented.

### 3.5. Control Layer

As the core of the control layer, the SDN controller includes the control function of the underlying device data plane, the internal collaborative management components for resource allocation and environment configuration, a virtualization component that provides network abstraction and policy enforcement for applications at the northbound interface, and a proxy component that reflects the resources and behaviors accessible to clients or applications. In general, the SDN controller should have the following functions:

- *Network Configuration and State Management*. It provides real-time monitoring and management of the network and corresponding configuration and maintenance according to network changes, such as statistical information, traffic information, and alarm information.
- *Data Storage Function*. The controller stores various network data for easy statistics and calls. For example, topology information, network status information, and traffic information.
- System Management Functions. It is responsible for the corresponding management functions of the operating system, such as resource allocation, initializing the operating environment, and system configuration.
- System Management Functions. It is responsible for the corresponding management functions of the operating system, such as resource allocation, initializing the operating environment, and system configuration.
- Interface Communication Function. The controller provides external applications with the ability to call abstract network resources and controller services through the northbound interface and completes the control of the underlying equipment through the southbound interface to realize the on-demand dynamic scheduling process of the network.

### 3.6. Data Layer

As a brand new network design concept, SDN has multiple implementations, but does not impose strict requirements on the form of data layer devices. SDN can be carried on traditional network equipment, such as hybrid switches; it can also be carried on new network equipment, such as OpenFlow switches. The ideal SDN emphasizes that the network is dominated by software. In this case, cheap, common, open, and standardized commercial hardware becomes the preferred bearer facility for SDN, which helps to reduce the total cost of network equipment. SDN separates the software and hardware of the data layer network equipment. Next, the data layer is introduced from the two aspects of network element hardware and middle software.

Network Element Hardware: network element hardware is now mostly concentrated in commercial hardware (COTS, commercial off-the-shelf products or commercial shelf products), which are commercial hardware products that follow open industry standards. Its biggest feature is universal, standard, low cost, better interoperability, and shorter design cycle and production cycle.

Intermediate Software: in the data layer, the software parts of network devices other than hardware and user applications are called intermediate software, including hardware drivers, network operating systems, and various open tools and management tools.

## 4. Data Resource Configuration

To optimize data resource allocation, one controller needs to be selected for each zone to manage. At this time, it is defined that *V*_*O*,*P*_ means that the area *Q*_*O*_ is connected to the controller *R*_*P*_. It is a binary variable, that is:

(1) $$\begin{array}{c} V_{o,p}=\left\{\begin{array}{cc} 1, & \text{Controller }R_{p}\text{ control area }Q_{o},\\ 0, & \text{Otherwise.} \end{array}\right. \end{array}$$

Recording selection strategy *V*=[*V*_*O*,*P*_]. Any zone has one and only one controller to control it, then:

(2) $$\begin{array}{c} \sum_{p\in R_{p}}V_{o,p}=1,\;\forall o\in Q_{o}. \end{array}$$

To maintain the normal operating speed of the network. It is not possible to overload any controller with:

(3) $$\begin{array}{c} \sum_{o\in Q_{o}}V_{o,p}a_{o}\leq K_{p},\;\forall p\in R_{p}, \end{array}$$

where *a*_*o*_ is the traffic volume of the area *o* and *K*_*P*_ is the maximum load of the controller *p*.

In addition, the deployment position of controller *R*_*P*_ is recorded as *W*_*O*,*P*_, indicating that controller *R*_*P*_ is deployed on area *Q*_*O*_, and there is

(4) $$\begin{array}{c} w_{o,p}=\left\{\begin{array}{cc} 1, & \text{Controller }R_{p}\text{ control area }Q_{o},\\ 0, & \text{Otherwise.} \end{array}\right. \end{array}$$

*C*_*o*,*h*_ is the distance between the two areas. To ensure the communication quality, the propagation delay should be less than the upper limit of the delay allowed by the system, then:

(5) $$\begin{array}{c} \frac{\sum_{h\in Q_{o}}V_{o,p}w_{h,p}c_{o,h}}{v\leq T_{\text{max}}},\;\forall o\in Q_{o},\;p\in R_{p}, \end{array}$$

where *v* is the data transmission rate and *T*max is the maximum propagation delay requirement of the network.

*U*_*o*,*h*_ is used to record whether two areas are controlled by the same controller, and matrix *U*=[*U*_*o*,*h*_] exists. Then, there are the following constraints:

(6) $$\begin{array}{c} U_{o,h}=\left\{\begin{array}{cc} 1, & \text{Controller control area }Q_{o}\text{ and area }Q_{h},\\ 0, & \text{Otherwise,} \end{array}\right.\\ \sum_{p\in R_{P}}V_{o,p}+V_{h,p}-1\leq u_{o,h},\;\forall o,h\in Q_{o}. \end{array}$$

*X*_*o*,*h*_ represents the number of times the user moves between areas *Q*_*o*_ and *Q*_*h*_, represented by matrix *X*=[*X*_*o*,*h*_]. Combining the above formula, the number of times that the SGW migrates (i.e., generates signaling overhead) during the frequent movement of the user can be calculated, which is denoted as *T*(*U*, *X*). Then, there is the following formula:

(7) $$\begin{array}{c} T\left(U,X\right)=\sum_{o\in Q_{o}}\sum_{h\in Q_{h}}x_{o,h}\left(1-u_{o,h}\right). \end{array}$$

The goal of this study is to deploy the location of the controller under the condition of meeting the communication indicators required by the user and formulate the control strategy between the controller and the area to reduce the signaling overhead between the controllers. Therefore, the mathematical model of the whole problem is as follows:

(8) $$\begin{array}{c} \min T\left(U,X\right),\\ Z1:\sum_{p\in R_{P}}V_{o,p}+V_{h,p}-1\leq u_{o,h},\;\forall o,h\in Q_{o},\\ Z2:\sum_{p\in R_{P}}V_{o,p}=1,\;\forall o\in Q_{o},\\ Z3:\sum_{o\in Q_{o}}V_{o,p}a_{o}\leq K_{p},\;\forall p\in R_{p},\\ Z4:\frac{\sum_{h\in Q_{o}}V_{o,p}w_{h,p}c_{o,h}}{v\leq T_{\max}},\;\forall o\in Q_{o},p\in R_{p},\\ Z5:V_{o,p}\in \left\{0,1\right\},\;\forall o\in Q_{o},p\in R_{p},\\ Z6:w_{o,p}\in \left\{0,1\right\},\;\forall o\in Q_{o},p\in R_{p},\\ Z7:u_{o,h}\in \left\{0,1\right\},\;\forall o\in Q_{o},h\in R_{h}. \end{array}$$

*Z*1 defines that any two zones are controlled by the same or different two controllers, and *Z*2 assigns a controller to each zone. *Z*3 and *Z*4 limit the capacity of the controllers in the network and the maximum propagation delay of the communication, respectively. *Z*5, *Z*6, and *Z*7 are all binary variables, which represent the distribution strategy between the controller and the region, the deployment location, and the control strategy between different regions.

The regional relevance matrix *M* of *G∗G* is constructed as follows:

(9) $$\begin{array}{c} M_{G*G}=\left(m_{o,h}\right)=\left[\begin{array}{cccc} m_{11} & m_{12} & ... & m_{1G}\\ m_{21} & m_{22} & ... & m_{2G}\\ \vdots & \vdots & \ddots & \vdots \\ m_{G1} & m_{G2} & \ldots & m_{GG} \end{array}\right]. \end{array}$$

It satisfies the following:

(10) $$\begin{array}{c} \sum_{o=1}^{G}m_{oh}=1,\;h\in Q_{h}. \end{array}$$

Element *m*_*oh*_ in matrix *M*_*G∗G*_ represents the transition probability of the user between region *o* and region *h*. The matrix is symmetric and has the following:

(11) $$\begin{array}{c} m_{oh}=m_{ho}. \end{array}$$

For any point *o*, its degree is the sum of the weights of all edges connected to it, namely:

(12) $$\begin{array}{c} c_{o}=\sum_{h=1}^{G}m_{oh}. \end{array}$$

Considering the actual host CPU performance, the data processing capability of the protocol function module is set to the level of several hundred thousand units per second. In addition, we set the network time limit in *μ*s. The specific simulation parameters are set as shown in Table 5.

Assume there are 10,000 users in the entire system, randomly distributed in 100 generated regions. The regional correlation matrix reflecting the user's movement habits is randomly generated, and the user moves between different regions once according to the roulette selection method of the matrix. Assuming that the number of controllers deployed in the network increases from 1 to 15, the relationship between the switching times between the controllers of the three algorithms is observed.  Figure 7 shows a diagram of the switching number of the user random mobile controller.

It can be seen from Figure 7 that with the increase in the number of controllers, when 10,000 users move randomly in adjacent areas, the switching times between the controllers of the two controller deployment strategies based on spectral clustering are significantly less than that of the random deployment controller strategy. From the algorithm analysis, the spectral clustering algorithm clusters the regions according to the similarity of the user's mobile behavior habits, which ensures that the regions under the same controller are highly correlated and the correlation between different controllers is low, so the deployment effect is better. So it can be concluded that, compared with the random deployment strategy, the controller deployment method based on spectral clustering reduces the number of handovers between controllers and reduces the signaling overhead of the system.

During this simulation, the system randomly generated 200 regions, and it was assumed that the maximum number of controllers deployed in the system was 8. 10,000 users are distributed in each region according to a randomly generated regional correlation matrix. The variance of the number of areas managed by the controller under different algorithms is compared, as shown in Figure 8.

Figure 8 shows that the variance between clusters of controller deployment strategies based on the RatioCut spectral clustering algorithm is the smallest, while the NCut spectral clustering performs slightly better than the random deployment method. When the number of controllers is small, the difference between the algorithms is very large; if the number of controllers increases, the performance difference between the three types of algorithms gradually decreases. We can conclude that RatioCut spectral clustering is the preferred algorithm to reduce the signaling overhead in the network and ensure load balancing between controllers.

Keeping other parameters unchanged, different regional topologies are randomly generated, and 10 controllers are always deployed in different network topologies. Observing the number of variances between controller clusters in different networks, the results are shown in Figure 9.

As can be seen from Figure 9, when the number of regions is small, the intercluster variance of the three deployment strategies is not much different, but when the number of regions gradually increases, the performance of the deployment strategy based on the RatioCut clustering algorithm is significantly better than the other two algorithms. Therefore, it can be concluded that in large-scale systems, the RatioCut clustering algorithm effectively ensures the load balance of the controller and improves the system performance.

Keeping other parameters unchanged, the arrival rate of user data flow takes a fixed value of *γ* = 50000. Assuming that user service requirements for the protocol are randomly generated, the relationship between the total number of protocol function modules required by the proposed algorithm and the benchmark algorithm and user service requests is observed, as shown in Figure 10(a). Assuming that the user's business requirements for the protocol are randomly generated, the relationship between the total number of protocol functional modules required by the two algorithms and the system time limit is observed, as shown in Figure 10(b).

Figure 10(a) shows that when the time limit of the system is fixed and the total number of service requests received is the same, the number of protocol function modules allocated by the GAA algorithm is 20% to 30% less than that of the RAA algorithm. So, it can be concluded that compared with the RAA algorithm, the GAA algorithm saves more network resources. Figure 10(b) shows that the GAA algorithm works better in a system with strict time limit and can greatly improve the utilization of network resources.

## 5. Discussion

The impact of controller deployment on network resources based on SDN technology is studied. This study mainly combines the behavioral habits of users under random movement to generate a base station correlation matrix based on user behaviors and habits and then uses the spectral clustering algorithm to cluster the base stations to complete the deployment of the controller; at the same time, a random user mobility model is established, and it is verified that in the EPC network, the spectral clustering algorithm SGW-C has fewer migrations in the process of frequent user mobility, thereby reducing the signaling overhead between controllers. This study analyzes and studies the allocation of protocol function modules under SDP technology, establishes the equivalent queuing theory model of the problem, and proposes an allocation algorithm through mathematical derivation, which realizes the rational allocation of network resources. Through simulation work, it is verified that the algorithm is better than the benchmark algorithm in terms of network resource consumption.

The construction of the macroeconomic management information system in XX Province provides information guarantee for the provincial party committee and the provincial government to accurately grasp the economic situation of the province, to ensure information flow and sharing, business coordination, and scientific decision-making among economic functional departments, further strengthening the government's macro-control and ability to respond to emergencies and to stabilize the market. Therefore, the project construction is absolutely necessary and urgent.

## 6. Conclusion

This study studies the deployment of control network elements in the system based on SDN technology. First of all, the functional network elements and interfaces in the system are introduced, and the SGW migration process in the user movement process is analyzed. Secondly, on the problem of minimizing signaling overhead in the process of frequent random movement of users in the system, we propose a controller deployment strategy based on a clustering algorithm in combination with the user's mobile behavior. Finally, a series of model simulations and system-level simulations are used to compare the advantages and disadvantages of the clustering algorithm and the benchmark algorithm. Aiming at the user's customized service request in SDP, the deployment idea of virtual protocol stack under SDP platform is proposed, and the related queuing theory model is given and deduced. Finally, according to the given queuing model, the allocation strategy of the functional modules of the SDP protocol is proposed and compared with the random allocation algorithm. The final simulation results show that in the time-limited network, the allocation algorithm is used to allocate fewer protocol function modules, which saves network resources and improves the resource utilization of the entire network. According to the actual situation of XX Province, this study builds a macroeconomic management information system, which provides certain help for improving work efficiency and increasing the accuracy and pertinence of data analysis. However, there are still some deficiencies in the actual construction and use process. For example, in the information acquisition stage, effective macroeconomic information cannot be quickly identified, and it still relies on artificial data screening and collection; in addition, failing to establish an effective connection with the big data analysis system, with the help of the power of big data analysis, the operating efficiency of the system can be further improved, but we still have reasons to believe that in the near future, the macroeconomic management information system can provide more effective help in economic development and socialist social construction.

## Figures and Tables

**Figure 1:** Diagram of information sharing.

**Figure 2:** Schematic diagram of business management information process.

**Figure 3:** Schematic diagram of the economic decision-making process.

**Figure 4:** Diagram of policy coordination and business synergy.

**Figure 5:** SDN network architecture sketch.

**Figure 6:** SDN architecture diagram.

**Figure 7:** User random movement controller switching number chart.

**Figure 8:** Controller intercluster variance comparison result 1.

**Figure 9:** Controller intercluster variance comparison result 2.

**Figure 10:** System simulation results.

**Table 1:** Basic support resource allocation list table.

Serial number	Equipment name	Basic layout	Quantity
1	Application system computing resources	CPU: 4pcs 8 cores	10 sets
		Memory: 256 GB	
		Hard disk: 300 GB X2	
		RAID level: RAID1	
		Network interface: gigabit network card interface X2, 2∗10 GE interface	
		HBA interface: 2∗8 Gb	
2	Database computing resources	CPU: 4pcs 8 cores	4 sets
		Memory: 256 GB	
		Hard disk: 600 GB X3	
		RAID level: RAID5	
		Network interface: gigabit network card interface X2,2∗10 GE interface	
		HBA interface: 2∗8 Gb	
3	Data exchange predecessor service server	Integration of existing resources	2 sets
4	Large-scale relational database software	Supports 30 million concurrent users	2 sets
		Supports multi-node redundancy	
		Oracle Enterprise Edition (RAC)	
5	Data exchange platform services ware	Integration of existing resources	1 set
6	Cloud service management center service server	Integration of existing resources	1 set
7	Virtualization management center services server	Integration of existing resources	1 set

**Table 2:** Database server computing power projection table.

Provincial access terminal	*z*1	500
Concurrent 1	*b*1	0.45
City and state access terminals	*z*2	4200
Concurrent 2	*b*2	0.1
District and county access terminals	*z*3	9050
Concurrent 3	*b*3	0.02
Transaction response time	*t*	5
*M*2	*M*2	9912
Number of database transactions per transaction	a	7
Ratio of benchmark TPC indicator values to actual transaction values	*M*0	15
Processor capacity margin	*M*1	0.3
TPC-C= (*M*2 × *a* × *M*0)/(1 − *M*1)		1486800

**Table 3:** Application server computing power projection table.

Provincial access terminal	*z*1	500
Concurrent 1	*b*1	0.45
City and state access terminals	*z*2	4200
Concurrent 2	*b*2	0.1
District and county access terminals	*z*3	9050
Concurrent 3	*b*3	0.02
Transaction response time	*t*	5
Average request service	*M*	165.2
Session request service	*M*2	214.76
Entity request transactions	*M*1	264.32
Benchmark business complexity	*G*	2.6
Processor capacity margin	*T*	0.3
Jops = (*M*1 + *M*2) × *G*÷(1 − *T*)		1779.44

**Table 4:** SDN controller deployment summary.

Serial number	Controller deployment objectives	Adoption of algorithms
1	Minimize average propagation delay	*K*-median clustering, normalized cut map
2	Minimize maximum propagation delay	*K*-center clustering, improved *K*-means clustering
3	Reduce network failure rate	Adding alternate paths and nodes, genetic algorithm
4	Increase network throughput	Cooperative optimization algorithm, hierarchical analysis method, dynamic allocation algorithm
5	Controller load balancing	Hierarchical cluster taxonomy
6	Reduce network overhead	Backpacking algorithm, simulated annealing algorithm, greedy algorithm

**Table 5:** Simulation parameter settings.

Simulation parameters	Simulation value	Simulation parameters	Simulation value
Network user request maximum	198	Reach of user data streams	10^5 − 9∗10^5
Number of SDP business types	6	SDP service site types	7
Capacity per SDP site	10^6 − 1.2∗10^6	System processing time delay threshold	*T*0 = 1.35 *μ*s, *T*1 = 1.19 *μ*s

## Data Availability

Data sharing is not applicable to this article as no new data were created or analyzed in this study.
